The article "Wearable Wireless Body Area Networks for Medical Applications" was retracted in 2023. Reasons: signs of a paper mill; suspected computer-generated content; unreliable results or conclusions; concerns about the data.

# Wearable Wireless Body Area Networks for Medical Applications

**DOI:** 10.1155/2021/5574376

**Published:** 2021-04-24

**Authors:** Carlos A. Tavera, Jesús H. Ortiz, Osamah I. Khalaf, Diego F. Saavedra, Theyazn H. H. Aldhyani

**Affiliations:** ^1^Universidad Santiago de Cali, Cali, Colombia; ^2^Closemobile R&D Telecommunications LS, Fuenlabrada, Spain; ^3^Al–Nahrain University, Bagdad, Iraq; ^4^Community College of Abqaiq, King Faisal University, P.O. Box 4000 Al-Ahsa, Saudi Arabia

## Abstract

In recent times, there has been a significant growth in networks known as the wireless body area networks (WBANs). A WBAN connects distributed nodes throughout the human body, which can be placed on the skin, under the skin, or on clothing and can use the human body's electromagnetic waves. An approach to reduce the size of different telecommunication equipment is constantly being sought; this allows these devices to be closer to the body or even glued and embedded within the skin without making the user feel uncomfortable or posing as a danger for the user. These networks promise new medical applications; however, these are always based on the freedom of movement and the comfort they offer. Among the advantages of these networks is that they can significantly increase user's quality of life. For example, a person can carry a WBAN with built-in sensors that calculate the user's heart rate at any given time and send these data over the internet to user's doctor. This study provides a systematic review of WBAN, describing the applications and trends that have been developed with this type of network and, in addition, the protocols and standards that must be considered.

## 1. Introduction

A WBAN is a network built with different intelligent elements such as sensors, nodes, and actuators. This network is designed to work on the human body and its surroundings. The elements that conform the network must be highly reliable, exhibit low consumption, be operational at a high range (maximum 5 m), must be resistant to interference, and must be able to operate within a wide range of transmission speeds [1]. These networks were first incepted in the 90s at Massachusetts Institute of Technology under the hypothesis of being able to attach electrical devices to the human body. Ever since, a high emphasis has been placed on increasing the bandwidth of the devices and consequently, decreasing their scope, consumption, and price.  Figure 1 below provides a comparison between a WBAN network and other networks [2].

### 1.1. Regulations

The current IEEE 802.15.6 standard for WBAN technologies was published in 2012, and it is “a standard for short-range wireless communication devices” located near or within the human body (although it may not be limited to just human beings). WBAN technologies use existing industrial, scientific, and medical (ISM) bands, as well as the different frequency bands endorsed by local doctors or regulatory authorities [3]. This standard considers the effects on portable antennas owing to the presence of a human being (this varies depending on whether it is a man, a woman, whether they are tall, or thin), and the radiation patterns required to reduce specific absorption rates (SAR) in the body and changes from characteristic personal movements.  Table 1 below shows the OSI model for a WBAN network [4].

Based on IEEE 802.15.6, the WBAN communication architecture is presented in Figure 2.

Within the regulations, there are some requirements that must be considered, as presented below [5–7]:

- Nodes must be removed and inserted into the network in less than 3 s
- Each WBAN must support 256 nodes
- Even if the person is constantly moving, the nodes must be able to provide stable and reliable communication
- System latency should be less than 125 ms for medical applications and less than 250 ms for nonmedical applications. Their fluctuation must be less than 50 ms
- WBANs on and within the body must be able to coexist within the same range. They must be supported on 10 randomly distributed WBANs and located in a physical layer in a 6 m^3^ cube
- A WBAN can incorporate the UWB technology with narrow band transmission to cover different environments and support high data rates
- They must also incorporate QoS management features to be self-correcting and secure and support priority services
- WBANs must also include energy-saving systems that will allow them to operate in power-restricted environments
- WBAN links must support transfer rates in a range from 10 Kb/s to 10 Mb/s
- The packet error rate (PER) for a 256-octet payload must be less than 10% for most links that are based on the best PER performance [8–12]
- All equipment must be capable of transmitting at 0.1 mW (−10 dBm). The maximum radiated transmit power must be less than 1 mW (0 dBm). This complies with the specific absorption rate (SAR) that the Federal Communications Commission has established, which is 1.6 W/Kg per each 1 g of body tissue
- They must be able to function in an environment where networks of different standards operate with each other to receive information

Table 2 below lists the frequency bands designated by the IEEE for WBAN [13, 14].

### 1.2. Applications

As applications can be categorized depending on the field in which the WBANs are involved, some applications range from military use to ubiquitous healthcare, training, sports, and entertainment. IEEE 802.15.6 has categorized applications of both medical and nonmedical nature.  Table 3 below contains this distribution and provides evidence that the main characteristics of all WBAN applications are aimed at improving user quality of life.

Within the existing literature, different WBAN healthcare applications were found.  Table 4 below describes some of these findings. The process implemented for searching, filtering, and selecting this information will be described in the methodology section.

### 1.3. WBAN Challenges

WBAN nodes are characterized by limited memory, processing, and power resources. Energy management is, as a matter of fact, considered an important challenge. As batteries are small and node power is limited, the energy consumption of the different devices needs to be reduced to secure a long battery life [30].

WBANs are important in the communication functionalities provided in medical applications and other application of smaller scope. Owing to their characteristics, some existing challenges and issues are discussed below.

Although WBANs allow a ubiquitous connection to the global network, they not only require support from the network infrastructure but also from different software implementations, such as remote procedures, database processing, and a user interface. Still, these implementations must feature low consumption and have little impact on the routing process [31].

Standards are still required for high-level data formats and which may also support using the user interface through social networks. The method and format used to deliver information outside the network are not usually implemented. Hence, the developer is responsible for the manner in which data are delivered to certain applications, implying that interoperability may be generated depending on the different solutions proposed [32, 33].

## 2. Methods

As part of the eligibility criteria, to conduct this systematic review, the following research question was taken into consideration: What are the different medical applications in which wearable WBAN technology is involved?

Bearing in mind this research question, the objective of this study was defined: to describe the different medical applications in which WBAN technology is involved.

Search sources: the bibliographic sources that were used to conduct this research are listed below:

1. IEEE
2. Springer
3. ScienceDirect

Search: having selected the topic and the databases, the systematic search was conducted, implementing the different keywords and their respective logical connectors. The keywords used and the ideal combination of logical connectors for subsequent implementation in the databases are listed below:

1. Sensor AND health AND WBAN
2. Sensor AND health AND “wireless body area network”
3. Sensor AND health AND (disease AND monitor AND microcontroller)

### 2.1. Selection

In this section, the different inclusion and exclusion criteria that were considered to filter the information are mentioned.

Inclusion criteria: the articles that should mainly be on the selected list are those that meet the following characteristics:

1. They must be in Spanish, English, or Portuguese
2. Articles must have publication dates no older than five years (2015–2020).
3. These must be downloadable articles
4. The main topic addressed by the authors must be linked to the wearable WBAN networks and their different implementations
5. The applications described by the authors must be oriented toward medical use in patients with different pathologies

Exclusion criteria: articles whose information are as follows:

1. Is not considered accurate or the author has not solved the research problem
2. The applications in which the WBAN is involved are not medical, but this technology is used as hobbies, laboratory practices, or to measure information that is not related to health

Bearing in mind this methodology, we started the exploration process, which lasted 31 days, and engaged the participation from three engineers. One of them is currently pursuing a Master's of computer science, and two of them hold PhDs in engineering. This consolidates the experience of the researchers to conduct the said research, with an odd number of researchers, for the correct choice of articles.  Table 5 shows the result of the different filters applied in the review.

As a result, Table 6 presents the wearable applications involving WBANs in health, the sensors used, and the characteristics considered by the authors.

In later sections, the results obtained from this exploration are presented.

## 3. Results and Discussions

From Table 7, a trend inclining toward the use of communication devices such as low-energy Bluetooth and WIFI can be observed owing to their great standardization and ability to connect to a mobile hub, such as those available in most smartphones. This can be attributed to the fact that most of the applications found used a hub, such as those available in most smartphones, because it allows the information to be directly loaded to a cloud service if necessary.

In addition, at the research level, there is a tendency to better guarantee the reliability of the data obtained through the sensors, as well as improving the consumption of the devices developed using techniques for energy saving, power generation, or even dedicated FPGA chips. Conversely, aspects such as security, communication reliability, and real time are less approached, and on the contrary, more challenges are generated for existing protocols for improvement or new models are constantly being proposed. It was found that 66% of WBAN wearable applications used Bluetooth, 17% WIFI, and only 3.5% ZigBee or NFC. The most common problems noted were heart problems and respiratory disorders.

Real-time applications were less widely used, commonly using protocols such as ZigBee. They have the disadvantage that they are limited to a local environment because switching to an internet protocol increases their latency. However, although wearable WBAN applications do not commonly use real time, information processing is performed through artificial intelligence to diagnose risk conditions and generate early medical alerts.

Bioimpedance and capacitance analysis were used as support in the diagnosis and monitoring of different pathologies because they analyze the body sections composition, evaluating in a general way the hydration status, lean, and fat mass. Even so, there are other applications that also involve this technique, for example, to make 3D images of internal organs to track diabetic patients. Conversely, inertial and ECG sensors were the most used in the different systems, being deemed as user-friendly sensors owing to their many user modules.

It is expected that with the development of new technological products such as smart watches and wireless headphones, which currently have a great impact on society, they will continue to improve the hardware related directly to the technologies used for WBAN. These devices have encouraged the improvement of technologies such as Bluetooth (Bluetooth 5.2) and low-power processors, improving the ability to connect to multiple nodes, reducing energy consumption, and ability to preprocess sensor data according to medical models, helping to guarantee the security and reliability of communications, as well as the improvement of transmission speeds, and in addition, to achieve future applications in real-time outside a local environment, through the development of technologies such as 5G and tactile internet.

## 4. Conclusion

WBAN technology is increasingly being used in applications where people and their well-being are involved, increasing the presence of technologies in patients' health. WBAN devices not only provide constant information about patients and their pathology but can also diagnose diseases and facilitate treatments and constant medical involvement.

It is important to continue advancing in the continuous reliability improvement of the information obtained using the WBAN, as well as device autonomy. This will allow the creation of new robust models, through techniques such as artificial intelligence that can provide permanent diagnosis and monitoring for diseases affecting a large part of the population, while taking advantage of the constant improvement of technologies such as tactile internet and personal gadgets.

## Figures and Tables

**Figure 1:** Comparison between WBAN and other networks.

**Figure 2:** WBAN communication architecture.

**Table 1:** OSI model for a WBAN.

Media access control and security		
Physical layer (PHY) narrow band (NB)	Ultrawide band (UWB)	Human body communications PHY (HBC)

**Table 2:** Table 2 is reproduced from Movassaghi et al. [15], [under the Creative Commons Attribution License/public domain [15]].

Human body communication	
Frequency	Bandwidth
16 MHz	4 MHz
27 MHz	4 MHz
Narrowband communication	
Frequency	Bandwidth
402–405 MHz	300 KHz
420–450 MHz	300 KHz
863–870 MHz	400 KHz
902–928 MHz	500 KHz
956–956 MHz	400 KHz
2320–2400 MHz	1 MHz
2400–2438.5 MHz	1 MHz
UWB communication	
Frequency	Bandwidth
3.2–4.7 GHZ	499 MHz
6.2–10.3 GHz	499 MHz

**Table 3:** WBAN applications according to IEEE 802.15.6.

WBAN applications			
Medical			Nonmedical
Wearable WBAN	Implantable WBAN	Remote control of medical devices	
Asthma. Portable health monitoring. (cardiovascular diseases, diabetes, and temperature).	Cancer screening. Cardiovascular diseases (CD).	Telemedicine systems. Security to uniformed personnel.	Entertainment applications. Emergencies (nonmedical).

**Table 4:** Different WBAN applications.

Reference	Aplicación	Contribution	Medical	
			Wearable WBAN	Remote control of medical devices
[16]	It uses Bluetooth communication to measure body temperature, heartbeats, and possible falls.	It implements power by solar energy.	x	
[17]	It uses a GSM module to send heartbeat and body temperature information.	Optical sensor.		x
[18]	Maintains constant measurement of different medical patient parameters.	System with first aid assistance instructions.		x
[19]	It uses an ARM7 to determine the patient's heart condition.	Uses the android platform to communicate the system with the doctor.		x
[20]	It measures the person's heart rate, blood pressure, temperature, and breathing.	It uses a GSM modem to send the information to the doctor.		x
[21]	Assesses patient vibrations to determine whether the patient suffers from Parkinson's disease (PD).	The system makes it possible to determine the evolution of the disease.	x	
[22]	It uses sensors on the cellular phone to analyze the patient's gait and determine if the patient suffers from PD.	Implement a smartphone, database, and web application.		x
[23]	It measures the kinematics of the patient's gait to determine if they have PD.	Implement sensors in the lower limbs and upper body.	x	
[24]	Sensors placed on the soles of the feet to determine whether the patient suffers from PD.	Mobile application was implemented to monitor the patient.	x	
[17]	Sensors in the lower body to determine whether the patient suffers from PD.	It uses ZigBee technology and protocols.	x	
[25]	Implementation of inertial sensors to determine whether the patient suffers from multiple sclerosis.	—	x	
[26]	EEG sensor for assessing different brain activities.	Uses ensemble classifier for epileptic seizure detection for imperfect EEG data.	x	
[27]	System for real-time detection of epilepsies.	The sensor medium access control (SMAC) protocol is used to reduce delays in the time for sending information.		x
[28]	Clock sensor for detecting epilepsies in real time.	—		x
[29]	Clock sensor for monitoring seizures in real time.	Implement communication through the cloud.		x

Implantable WBANs and nonmedical applications were not considered.

**Table 5:** Summary of filtered articles.

	Keywords	Year and type filter	Title	Abstract	Chosen
IEEE	750	572	84	76	18
Springer	2,415	678	51	40	10
ScienceDirect	1,107	900	34	10	6
				Total	34

**Table 6:** Wearable WBAN applications in health.

Reference	Sensors used	Pathology or type of measurement	Communication method	Sensor reliability	Errors when sending data	Security	Energy saving	Real-time
[34]	Biompedance	Chronic kidney disease	Bluetooth	X				
[35]	MEMS inertial sensors [35]	Osteoporosis, osteoarthritis, dementia, Alzheimer's, Parkinson's	Bluetooth	X				
[36]	Heart sound sensor	Cardiovascular disease (CD)	Bluetooth 4.0	X				
[37]	Flow, accelerometer, microphone, strain, skin impedance, ECG, pulse, VOC, ozone, humidity/temp	Chronic respiratory disease	BLE	X			X	
[38]	ECG, accelerometer [38]	CD	NFC	X		X		
[39]	ECG signal monitoring	CD	Bluetooth 4.0	X				
[40]	Capacitive electromyography (CEMG)	Chronic inflammatory myopathies	Wire	X				
[41]	Microsoft Band [41]	Autonomic Dysreflexia (AD)	Bluetooth	X				
[42]	Inertials and carbon dioxide concentration detection device	Respiratory disorders	Wire					
[43]	Inertials, magnetometer	PD	Bluetooth					
[44]	Any ECG sensor	Cardiac care	Bluetooth/wifi/3G	X				X
[45]	Near infrared spectroscopy (NIRS)	Cerebral vascular diseases (CVDs)	Bluetooth	X				
[46]	ECG	CD	BLE				X	
[47]	ECG	Sleep apnea	BLE	X			X	
[48]	Light-based sensor	Daily blood pressure measurement	WIFI			X		
[49]	Humidity capacitance	Irregular respiratory diseases	Bluetooth	X				
[50]	Heart rate, temperature sensor, pressure	Physical parameters	WIFI			X		
[51]	Photoplethysmogram (PPG), ECG	Arising heart disease and stroke or any emergency condition	WIFI			X		
[52]	ECG, accelerometer Gyroscope Magnetometer	Sleep apnea syndrome (OSAS)	Bluetooth low energy (BLE)	X				
[53]	Heart rate, temperature, blood pressure	Continuous supervision	Bluetooth	X	X		X	
[54]	Pressure system	Chronic venous disorder	Bluetooth	X				
[55]	Measurement units	Breathing frequency monitoring	BLE				X	
[56]	ECG	Long-term homecare	ZigBee	X			X	
[57]	Inertial sensors	Home monitoring of motor fluctuations in PD	BLE	X				
[58]	ECG	Telemonitoring and cloud	NRF24L01		X			X
[59]	EMG device	Masticatory muscle activity	BLE	X				
[60]	Pulse oximetry	Sleep apnea detection	WIFI/Bluetooth	X			X	

**Table 7:** WBAN trends.

Reference	Application	Novelty	Sensors
[61]	Long-term continuous medical monitoring	Autonomous system, by means of solar energy	Inertials, temperature, and pulse
[62]	PD	Holistic system	Microsoft band, speech analysis, finger tapping
[63]	Classification of physical activity	Classification method using smartphones	Inertial
[64]	Peripheral artery disease	Passive wearable skin patch sensor measures	Electromagnetic resonant sensor
[65]	Detection of abnormalities, as well as intrusions, such as forgery, insertions, and modifications in the ECG data	Identify anomalies in ECG signals	Dataset
[66]	Proposal for emergency classification transmission	Priority data transmission	Oxygen in blood, pulse, and position measurements
[67]	Stroke, PD, and epilepsy	Garment with integrated sensors, user needs such as design and comfort are identified	Accelerometer, gyroscope, and ECG

## Data Availability

The data is available in https://www.gambitcomm.com/site/gambit4.shtml?gclid=Cj0KCQiAx9mABhD0ARIsAEfpavTHRH-mpys3ZJQbOuSmjUcvhz-wV5kl4-2l6-t5WQwF2DacULvftCgaAvXqEALw_wcB.
